The article "Risk Factors and Prognostic Analysis of Gastrointestinal Stromal Tumor Recurrence-Metastasis" was retracted in 2023. Reasons: signs of a paper mill; suspected computer-generated content; unreliable results or conclusions; lack of ethics approval or compliance.

# Risk Factors and Prognostic Analysis of Gastrointestinal Stromal Tumor Recurrence-Metastasis

**DOI:** 10.1155/2022/1127146

**Published:** 2022-07-18

**Authors:** Shan Chen, Kanru Sang, Wenjing Chen, Jinji Jin, Xiaolei Chen, Guanbao Zhu, Pengfei Wang, Yiqi Cai

**Affiliations:** ^1^First Clinical College of Wenzhou Medical University, Wenzhou, China; ^2^Department of Gastrointestinal Surgery, The First Affiliated Hospital of Wenzhou Medical University, Wenzhou, China

## Abstract

**Objective:**

Gastrointestinal stromal tumors (GISTs) are potential malignancies that occur in the digestive tract. This study aimed to investigate the risk factors and prognosis of recurrence and metastasis of gastrointestinal stromal tumor (GIST).

**Methods:**

From January 2018 to December 2019, 422 patients with GIST who received surgery in the First Affiliated Hospital of Wenzhou Medical University were enrolled. Their clinical data were retrospectively analyzed, and their follow-ups were continued until March 31, 2022. Subsequently, univariate and multivariate Cox analyses, survival curves, and nomograms were adopted to explore the relationship between clinicopathological characteristics and recurrence or metastasis in patients with GIST.

**Results:**

Univariate and multivariate Cox analysis exhibited that the prognosis of patients was affected by tumor rupture (*P* = 0.040), tumor location (*P* < 0.001), tumor diameter (*P* = 0.016), mitotic figures (*P* < 0.001), and risk grade (*P* < 0.009). The above variables were selected to create the nomogram for 3-year disease-free survival (DFS). The 3-year the ROC (receiver operating characteristic) curves of the nomogram were (0.878 95% confidence interval [CI]: 0.871–0.939).

**Conclusion:**

Collectively, risk factors affecting postoperative recurrence or metastasis of GIST consist of primary site of tumors, tumor rupture, tumor diameter >10 cm, high-risk tumor classification, and mitotic figures ≥10 per 50 HPFs. And the application of nomogram may help physicians provide individualized diagnosis and treatment for patients with GISTs following surgical resection.

## 1. Introduction

Gastrointestinal stromal tumor (GIST) is a rare tumor arising from the gastrointestinal tract, with an incidence of 0.1%–3% of all gastrointestinal malignancies [1]. However, in gastrointestinal tract, GIST is the most common mesenchymal tumor [2] and small intestinal malignant tumor, affecting 10-20 people per million [3]. Notably, GIST shows an increasing trend to its incidence in recent years [4]. GIST originates from interstitial cells of Cajal and their stem cells, and their mainly histological types enroll spindle, epithelioid, and mixed cells. The dominating biological characteristics of GIST are KIT gene (75%) activation or PDGFR*α* gene (15%) mutations, which result in continuous activation of tyrosine kinase receptors and continuous proliferation of tumor cells [5]. In addition, 50% to 70% GIST occur in the stomach (70% in the body of stomach, 15% each in the antrum and cardia), 30% in the small intestine, and occasionally in other parts of the abdominal cavity (colon, rectum, appendix, esophagus, and liver) [6].

The article "Risk Factors and Prognostic Analysis of Gastrointestinal Stromal Tumor Recurrence-Metastasis" was retracted in 2023. Reasons: signs of a paper mill; suspected computer-generated content; unreliable results or conclusions; lack of ethics approval or compliance.

The clinical manifestations of GIST lack specificity, so its diagnosis largely relies on imaging tests and pathological biopsy [7]. Despite adopting complete surgical resection as a mainstay treatment for localized and primary GIST [8], the 5-year recurrence rate of patients after treatment is estimated as high as 29.5% [9]. At present, important independent factors predicting GIST recurrence include the tumor mitotic rate, size, location, and tumor rupture [10], and postoperative adjuvant tyrosine kinase inhibitor (TKI) treatment may delay recurrence [11]. Therefore, an evaluation of the recurrence and progression risks of GIST has become more and more important for patients; also, an exploration to additional prognostic factors of recurrence risk stratification might increase the prognostic accuracy [12].

In this study, we analyzed the risk factors of metastasis and recurrence in patients with GIST. Specifically, nomograms were plotted with 3-year disease-free survival (DFS) to provide theoretical guidance for individualized postoperative prognosis analysis and intervention. And area under the curve (AUC) of nomograms reached 0.878 (95% confidence interval [CI]: 0.871–0.939), indicating that the reliability of clinical use was relatively strong.

## 2. Materials and Methods

### 2.1. General Information

A total of 422 patients diagnosed with GIST in the First Affiliated Hospital of Wenzhou Medical University from January 2018 to December 2019 were included in this study. Baseline data and clinical characteristics of patients were recorded. This study was a retrospective analysis requiring no informed consent, and all procedures were approved by the Ethics Committee of the First Affiliated Hospital of Wenzhou Medical University.

Inclusion criteria: (1) the age of patients ≥ 18 years; (2) with the primary tumor diagnosed in 2018-2019, and regular chemotherapy drugs for GIST were used according to the guidelines of the Chinese Society of Clinical Oncology (CSCO) [13, 14]. And there were no cases of preoperative neoadjuvant therapy in the included patients; (3) with GIST confirmed by test results of biopsy specimens which were obtained during laparotomy or laparoscopic, endoscopic resection; (4) complete outpatient/emergency follow-up data could be obtained after surgery. The exclusion criteria were as follows: (1) primary tumor occurring before 2018, and recurrent tumor occurring in 2018-2019; (2) confirmed as leiomyoma, fibroma, and other nonstromal tumors by intraoperative immunohistochemical results; and (3) lost to follow-up cases.

The article "Risk Factors and Prognostic Analysis of Gastrointestinal Stromal Tumor Recurrence-Metastasis" was retracted in 2023. Reasons: signs of a paper mill; suspected computer-generated content; unreliable results or conclusions; lack of ethics approval or compliance.

### 2.2. Relevant Indicators of Risk Stratification of Gastrointestinal Stromal Tumors

According to the modified National Institutes of Health (NIH) classification proposed by Joensuu in 2008 [15], patients with GIST were classified as very low risk, low risk, intermediate risk, and high risk (Table 1).

### 2.3. Disease-Free Survival

After surgery, patients with GIST were followed up for 36 months, and the prognosis and disease-free survival (DFS) were recorded. To be specific, follow-up was conducted in the outpatient clinic or by telephone, and the follow-up duration was calculated from the date of surgery to the date of finding recurrence and metastasis. Besides, patient prognosis included whether recurrence and metastasis occurred, and the site of tumor recurrence and metastasis, and DFS included the time from initiation of treatment to recurrence or metastasis of GIST. By the way, all data were finally censored at the last follow-up for the living patients.

### 2.4. Statistical Analysis

SPSS 26.0 statistical software was used for data analysis. Enumeration data were expressed as *n* (%); *χ*^2^ test was adopted for statistical analysis; measurement data were expressed as mean ± standard deviation (SD); and *t*-test was applied for statistical analysis. Univariate and multivariate Cox regression was performed to analyze the factors of tumor recurrence and metastasis. Survival curves were plotted using the Kaplan-Meier method, and nomograms of associated risk factors were generated using the R language. The receiver operating characteristic (ROC) analysis was used to evaluate the predictive ability of the nomogram of risk stratification systems. *P* < 0.05 served as the criterion of significant difference.

## 3. Results

### 3.1. General Clinical Data

Among 422 included patients, 199 (47.2%) were male, and 223 (52.8%) were female, aged from 25 to 82 years. Baseline data of patients are shown in Table 2. And in this paper, 12 patients suffered postoperative recurrence, with stomach as the common site; 31 patients had metastasis, with the liver as the common site (Table 3).

### 3.2. Correlation of Primary Tumor Location with Clinical Symptoms

To provide guidance for clinical diagnosis of GIST, 2 patients with multiple primary tumors were excluded, and the relationship between the chief complaints of the remaining 420 patients with GIST and their primary tumor sites was explored in this study. According to the results, a significant difference was identified in the complaints among patients with different primary sites (*P* < 0.001). Primary tumors in the stomach and other sites were mainly discovered by physical examination, and those in the small intestine presented with gastrointestinal bleeding (Table 4).

The article "Risk Factors and Prognostic Analysis of Gastrointestinal Stromal Tumor Recurrence-Metastasis" was retracted in 2023. Reasons: signs of a paper mill; suspected computer-generated content; unreliable results or conclusions; lack of ethics approval or compliance.

### 3.3. Analysis of Factors Associated with Recurrence-Metastasis in Patients with Gastrointestinal Stromal Tumors

#### 3.3.1. Recurrence-Metastasis Is Not Related to Blood Tumor Markers in Patients with Gastrointestinal Stromal Tumors

A total of 44 patients with GIST had tumor metastasis or recurrence during follow-up at 36 months after surgery. To investigate the relationship between postoperative metastasis or recurrence and blood tumor markers, patients were divided into recurrence-metastasis group (*n* = 36) and nonrecurrence-metastasis group (*n* = 386). Relationship between five blood tumor parameters and postoperative recurrence-metastasis in patients with GIST is displayed in Table 5. And there were no statistically significant differences in the five blood tumor indicators carcinoembryonic antigen (CEA, *P* = 0.405), alpha-fetoprotein (AFP, *P* = 0.459), cancer antigen 199 (Ca199, *P* = 0.461), Ca125 (*P* = 0.732), and Ca153 (*P* = 0.147) between the two groups.

#### 3.3.2. Correlations of Recurrence-Metastasis with Clinicopathological Characteristics in Patients with Gastrointestinal Stromal Tumors

To further investigate the relationship between recurrence-metastasis and clinical characteristics in patients with GIST, univariate and multivariate Cox regression analysis was performed. The results of univariate analysis suggested that postoperative recurrence and metastasis were closely correlated with tumor rupture, primary tumor site, tumor size, mitotic count, and risk classification (*P* < 0.05), but not with age, gender, body mass index, drinking, smoking, presence of gastrointestinal bleeding, presence of malignant tumors, and Ki-67 (*P* > 0.05). Further results of multivariate analysis showed that tumor rupture, primary tumor site, tumor size, mitotic count, and risk classification were independent risk factors for recurrence or metastasis of GIST (*P* < 0.05) (Table 6). After that, nomograms were plotted to qualify and analyze the effect of independent risk factors on prognosis. As shown in Figure 1, for patients with the primary site of tumors in the stomach, the tumor diameter ≤ 2 cm, the mitotic count ≤5 per 50 HPFs, the risk stratification as low/intermediate, and without tumor rupture, the 3-year DFS rate is higher than 90%, and the prognosis is better. By contrast, for patients with tumor rupture, nongastric primary site, tumor diameter>10 cm, mitotic count >10 per 50 HPFs, and high-risk grade, their total score was 290 points, and the 3-year DFS rate was less than 40%. ROC analysis for 3-year prognostic accuracy of the nomogram was performed, and according to the results, the 3-year AUC was nomogram, 0.878 (95% CI: 0.871–0.939).

The article "Risk Factors and Prognostic Analysis of Gastrointestinal Stromal Tumor Recurrence-Metastasis" was retracted in 2023. Reasons: signs of a paper mill; suspected computer-generated content; unreliable results or conclusions; lack of ethics approval or compliance.

#### 3.3.3. Survival Curve Analysis of the Correlation between Recurrence-Metastasis and Clinicopathological Characteristics in Patients with Gastrointestinal Stromal Tumors

Further survival curve analysis showed that different mitotic count (*P* < 0.0001), the presence of tumor rupture or not (*P* = 0.0003), risk classification (*P* < 0.0001), tumor location (*P* = 0.0006), and tumor diameter (*P* < 0.0001) all affect DFS in patients with GIST (Figure 2). To be specific, at 36 month-followed up, the DFS rate was 98.383% in patients with mitotic count <5 per 50 HPFs, 87.369% in patients with 5 per 50 HPFs ≤ mitotic count <10 per 50 HPFs and 66.757% in patients with mitotic count ≥10 per 50 HPFs (Figure 2(a)). And the DFS rate was significantly higher in patients without tumor rupture (96.838%) compared with that of patients with tumor rupture (86.475%) (Figure 2(b)), and much higher in low-risk–intermediate-risk patients (96.838%) compared with that in high-risk patients (83.769%) (Figure 2(c)). Also, patients with primary tumor site in the stomach had higher DFS rate (96.109%) than those in the nonstomach (87.389%) (Figure 2(d)). Additionally, the DFS rate was 98.383% in patients with tumor diameter ≤2.0 cm, 97.633% in those with 2.0 cm < tumor diameter ≤5.0 cm, 77.856% in those with 5.0 cm < tumor diameter ≤ 10.0 cm, and 87.500% in those with tumor diameter >10.0 cm (Figure 2(e)).

## 4. Discussion

In spite of the occurrence at any age, GIST is more common in adults, and the median age ranges from 60 to 65 years [16]. A survey and analysis from America showed that the incidence of GIST was similar in men and women [17]. In our study, the median age of patients was 60 years old, with a male-to-female prevalence ratio of 1 : 1.12, in line with previous literature reports.

The primary site of most mesenchymal tumors is in the stomach (60%–65%), followed by the small intestine (20%–30%), rare in the rectum, colon, and esophagus [18]. Besides, some studies have reported primary GIST in the liver [19]. As for mesenchymal tumor patients in our study, there were 298 patients whose primary site in the stomach (70.9%), 93 patients in the small intestine (22.1%), and 29 patients in other sites (6.9%), and two cases had multiple primary tumor. The primary tumor site was associated with the risk of the tumor. Under the condition of tumor diameter of 2.1–5.0 cm and 6–10 mitoses per 50 HPFs, the tumor with primary site in the stomach was graded as intermediate risk and that in nongastric primary tumor was graded as high risk. In this paper, univariate and multivariate Cox regression analysis showed that tumor rupture, tumor site, tumor size, and mitotic count were independent risk factors for recurrence or metastasis of GIST (*P* < 0.05). After predicting prognosis using nomogram, the score difference could reach 20 points between patients with primary tumor in the stomach and those in the small intestine, suggesting that patients with nongastric primary site (small intestine) had a higher risk of recurrence and metastasis. Gender is also an important risk factor affecting the prognosis of mesenchymal tumors [5]. Patryk Zemaca et al. concluded that male patients had a lower survival rate regardless of age [20]. Most of patients with mesenchymal tumors have no obvious symptoms, especially for GIST less than 1 cm in diameter, and the autopsy rate can reach 25% [21]. Most patients with mesenchymal tumors less than 2 cm in diameter are diagnosed by endoscopy, while larger GIST can invade blood vessels, and patients are usually accompanied by gastrointestinal bleeding and other clinical symptoms [22]. In our study, the first three reasons for hospital visits were physical examination, abdominal discomfort, and gastrointestinal bleeding, basically in line with the characteristics of mesenchymal tumors. In addition, some cases have perianal discomfort, nausea, anemia, and other clinical manifestations. Gastrointestinal bleeding was the main reason for patients with primary GIST in the small intestine to visit the hospital, while physical examination was the main reason for those with primary GIST in the stomach, and a correlation could be suspected between the primary tumor site and clinical symptoms. For patients with gastrointestinal bleeding, if mesenchymal tumor is suspected, but the tumor lesions cannot be discovered by gastroscopy and colonoscopy, the possibility of small intestinal GIST should be considered. Mesenchymal tumor located in small intestine has higher risk of recurrence or metastasis, and segmental intestinal resection is recommended to obtain negative resection margins [9, 23]. Imatinib, a preferred chemotherapeutic drug [22], can help advanced GIST patients obtain longer DFS and prevent metastatic adverse events when applied as adjuvant radiotherapy [24]. Unfortunately, given the limited number of samples and observation time in this study, it keeps unknown whether gastrointestinal bleeding is related to the clinical manifestations at the time of recurrence and metastasis of GIST.

The article "Risk Factors and Prognostic Analysis of Gastrointestinal Stromal Tumor Recurrence-Metastasis" was retracted in 2023. Reasons: signs of a paper mill; suspected computer-generated content; unreliable results or conclusions; lack of ethics approval or compliance.

The results of the nomogram in this study showed that the total score was 290 points and the 3-year DFS rate was less than 40% for patients with tumor rupture, nongastric primary site, tumor diameter >10 cm, mitotic count >10 per 50 HPFs, and high-risk grade. Additionally, survival curve analysis exhibited that different mitotic count (*P* < 0.0001), tumor rupture (*P* = 0.0003), risk classification (*P* < 0.0001), tumor location (*P* = 0.0006), and tumor diameter (*P* < 0.0001) all affected DFS in patients with GIST. Generally, the diameter of GIST ranges from 0.6 to 25.5 cm, with an average diameter of 8.78 ± 5.6 cm and a median diameter of 6.8 cm; however, giant GIST with a diameter of 34 cm have also been reported [25]. Therefore, some studies have selected 10 cm as the cut-off value affecting the prognosis [26]. Miettinen et al. believed that GIST with a diameter of more than 10 cm had a higher risk of recurrence and metastasis [27]. In our study, the diameter of GIST was 0.2–23 cm, with a median diameter of 4 cm. Among the 36 cases with recurrence and/or metastasis, 19.4% patients (7/36) had a tumor diameter of more than 10 cm. Nevertheless, among the cases without recurrence and metastasis, only 6.5% (25/386) had a diameter of more than 10 cm.

Mitotic count is considered to be the most powerful predictor of recurrence and metastasis of GIST [20, 27]. According to our analysis, the mitotic count greater than 5 per 50 HPFs accounted for 61.1% (22/36) of the recurrent and/or metastatic cases, with a statistically significant difference compared with that of nonrecurrent and metastatic cases [14.5% (56/386)]. Mitotic count is positively correlated with tumor volume, which affects the malignant potential of tumors together [20]. Univariate and multivariate Cox regression analysis showed that the mitotic count was an independent risk factor for recurrence or metastasis of GIST, and nomogram and survival curve analysis also revealed that the more mitoses, the smaller the 3-year DFS rate of GIST.

The common sites of metastasis of GSIT are liver, abdominal cavity, and lymph nodes [16, 19]. In the study by Jnmniensuk et al., the metastasis of GIST also mainly occurred in liver and abdominal cavity, but some other articles have also reported bone metastasis [28]. In our study, the liver and abdominal cavity are the most common metastasis sites, occasionally with bone and pleural metastasis, suggesting that attention is needed to be paid on the possibility of extraperitoneal metastasis of GIST in clinical practice. In addition, this study revealed that postoperative recurrence-metastasis in patients with GIST was not related to blood tumor markers. Tumor rupture is an independent evaluation indicator of GIST and is closely related to recurrence and metastasis. The rupture caused by endoscopic biopsy or intraoperative resection easily induces tumor metastasis, and some patients with malignant ulcers should be alert to the possibility of tumor rupture and metastasis [29]. When the primary tumor ruptures spontaneously or due to surgery, the tumor can be metastasized to the retroperitoneum, and then, retroperitoneal mesenchymal tumors can be formed. Terribly, the traditional treatment methods, such as surgical resection, radiotherapy, and systemic chemotherapy, have little effect on retroperitoneal mesenchymal tumors, and patients have a poor prognosis [9]. Of the 10 patients with rupture outside gastrointestinal tract, 8 cases suffered recurrence and metastasis, including 5 cases of abdominal metastasis, in our study. Such results indicated that tumor rupture could increase the risk of metastasis; therefore, endoscopy and surgical procedures should be performed with caution to avoid tumor dissemination caused by iatrogenic factors.

The article "Risk Factors and Prognostic Analysis of Gastrointestinal Stromal Tumor Recurrence-Metastasis" was retracted in 2023. Reasons: signs of a paper mill; suspected computer-generated content; unreliable results or conclusions; lack of ethics approval or compliance.

Some limitations can be observed in this study. Firstly, this is a single-center retrospective study on GIST patients receiving surgical treatment, and the conclusion obtained still needs to be validated by a prospective and appropriately designed study. Secondly, follow-up in this study is not sufficient. On the one hand, follow-up duration is short; on the other hand, only 3-year DFS after surgery has been recorded. And both follow-up time and DFS of patients need to be prolonged. Thirdly, due to the small sample size, a detailed stratified analysis of GIST patients has not been performed in this paper; therefore, a large-scale multicenter trial must be conducted to validate our scoring system before adopting the system in routine practice.

## 5. Conclusion

There is a certain correlation between the primary site of GIST and the clinical manifestations of patients. Postoperative recurrence-metastasis in the patients is not associated with blood tumor markers, but closely with primary tumor site, tumor rupture, tumor risk grade, and mitotic figures. Therefore, individualized diagnosis and treatment for GIST should be performed based on clinicopathological characteristics and prediction of the risk of postoperative recurrence and metastasis.

## Figures and Tables

**Figure 1:** Nomogram of statistically significant variables in multivariate Cox proportional hazards model. (a) Nomogram of statistically significant variables in multivariate Cox proportional hazards model: (1) rupture: 1; intraluminal rupture of digestive tract; 2 extraluminal rupture of digestive tract; (2) site: 0; no gastric; 1, gastric; (3) size: 0, ≤2.0; 1, 2.1-5.0; 2, 5.1-10.0; 3, >10.0; (4) mitotic index (per 50 HPFs): 1, ≤5; 2; 6-10; 3, >10; (5) classification of risks: 0, low/intermediate; 1, high. (b) Receiver operating characteristic curves for risk model to predict the PFS of patients with GISTs.

The article "Risk Factors and Prognostic Analysis of Gastrointestinal Stromal Tumor Recurrence-Metastasis" was retracted in 2023. Reasons: signs of a paper mill; suspected computer-generated content; unreliable results or conclusions; lack of ethics approval or compliance.

**Figure 2:** Kaplan–Meier survival curves for RFS of patients with gastrointestinal stromal tumors. (a) Mitotic count (group A: mitoses <5 per 50 HPFs; group B: 5 per 50 HPFs ≤ mitoses <10 per 50 HPFs; group C: mitoses ≥5 per 50 HPFs). (b) Tumor rupture (group A: no rupture; group B: with rupture). (c) Risk classification (group A: low risk-intermediate risk; group B: high risk). (d) Tumor location (group A: nonstomach; group B: stomach); (e) Tumor diameter (group A: tumor diameter ≤ 2.0 cm, group B: 2.0 cm < tumor diameter ≤5.0 cm; group C: 5.0 cm < tumor diameter ≤ 10.0 cm; group D: tumor diameter>10.0 cm).

**Table 1:** Risk stratification of gastrointestinal stromal tumors.

Risk stratification	Tumor diameter(cm)	Mitotic count (per 50 HPFs)	Primary location of tumor	The number of cases
Very low	<2.0	≤5	Any location	152
Low	2.1-5.0	≤5	Any location	119
Intermediate	2.1-5.0	>5	Gastric	44
	<5.0	6-10	Any location	
	5.1-10.0	≤5	Gastric	
High	Any size	Any mitotic rate	Tumor rupture	107
	>10.0	Any mitotic rate	Any location	
	Any size	>10	Any location	
	>5.0	>5	Any location	
	2.1-5.0	>5	Nongastric	
	5.1-10.0	≤5	Nongastric	

Note: HPF, high-power field.

**Table 2:** Baseline data of patients.

Item	Category	n (%)
Gender	Male	199 (47.2%)
	Female	223 (52.8%)
Age (year)		25-82 (median: 60)
	<60	205
	≥60	217
Smoking history	Yes	84
	No	338
Drinking history	Yes	86
	No	336
Body mass index	<18.5	14
	18.5–23.9	167
	>23.9	167
	Not detected	74
Accompanied by malignant tumors #	Yes	76
	No	346
Primary location of tumor	Stomach	298 (70.9%)
	Small intestine	93 (22.1%)
	Other locations	29 (6.9%)
	Multiple primaries	2 (0.5%)
Pathological results	≤5 per 50 HPFs	337
	> 10 per 50 HPFs	29
	Not detected	56
Tumor diameter		0.2–23 cm (median: 4 cm)
Immunohistochemical results	CD117-positive	93.4% (394/422)
	CD34-positive	90.8% (383/422)
	DOG-1-positive	93.1% (393/422)
	Ki-67-positive	81.75% (345/422)
Other parameters	S-100	5.7%(24/422)
	SMA	19.4%(82/422)
Risk stratification	Very low	152
	Low	119
	Intermediate	44
	High	107
Treatment method	Laparotomy	161
	Laparoscopic resection	133
	Endoscopic resection	128
Follow up results	Recurrence	5
	Metastasis	24
	Recurrence and metastasis	7
	No recurrence or metastasis	386

Note: # accompanied by malignant tumors such as gastric adenocarcinoma, primary malignant tumor of liver, and colorectal malignant tumor.

The article "Risk Factors and Prognostic Analysis of Gastrointestinal Stromal Tumor Recurrence-Metastasis" was retracted in 2023. Reasons: signs of a paper mill; suspected computer-generated content; unreliable results or conclusions; lack of ethics approval or compliance.

**Table 3:** Postoperative recurrence-metastasis location and proportion of patients with gastrointestinal stromal tumors.

Recurrence-metastasis location	Number of cases (*n*)	Proportion (%)
*Recurrence location*		
Stomach	5	41.6
Small intestine	2	16.7
Abdominal and pelvic cavity	2	16.7
Colon and rectum	2	16.7
Anal canal	1	8.3
Total	12	100%
*Metastasis location*		
Liver	11	35.4
Abdominal and pelvic cavity	9	29.0
Bone	1	3.2
Pleura	1	3.2
Multiple	9	29.0
Total	31	100%

**Table 4:** Primary tumor location and chief complaints.

Location	Physical examination	Abdominal discomfort	Gastrointestinal bleeding	Others	Total
Cardia	4	9	1	2	16
Fundus	45	40	5	3	93
Body	37	22	2	17	78
Greater curvature	22	11	4	3	40
Lesser curvature	22	11	8	4	45
Antrum	11	8	3	1	23
Other parts of stomach	0	0	0	3	3
Total (stomach)	141	101	23	33	298
Small intestine	23	25	30	15	93
Others	13	7	3	6	29

**Table 5:** Relationship between five blood tumor parameters and postoperative recurrence-metastasis in patients with gastrointestinal stromal tumors.

Blood tumor markers	Nonrecurrence-metastasis group (*n* = 378)	Recurrence-metastasis group (*n* = 44)	*P* value
CEA	1.35 (0.20-49.80)	1.20 (0.30-8.00)	0.405
AFP	2.47 (0.89-19.22)	2.84 (0.99-6.56)	0.459
Ca199	6.00 (0.80-625.8)	5.20 (0.80-43.80)	0.461
Ca125	7.90 (1.70-279.10)	12.00 (5.60-55.70)	0.732
Ca153	6.35 (2.10-23.60)	6.40 (2.80-13.00)	0.147

Note: CEA: carcinoembryonic antigen; AFP: alpha-fetoprotein; Ca: cancer antigen.

**Table 6:** Univariate and multivariate COX regression analysis of recurrence and metastasis in patients with gastrointestinal stromal tumors.

	Total (*N*)	Nonrecurrence-metastasis group (*n* = 386)	Recurrence-metastasis group (*n* = 36)	Univariate analysis		Multivariate analysis	
				Hazard ratio (95% CI)	*P* value	Hazard ratio (95% CI)	*P* value
Age	422			1.266 (0.646-2.480)	0.493		
≤60		190	15				
>60		196	21				
Gender	422			1.999 (0.994-4.021)	0.052		
Male		178	21				
Female		208	15				
BMI	381			0.727 (0.392-1.349)	0.312		
<18.5		12	2				
18.5-23.9		183	17				
>23.9		154	13				
Drinking history	420			0.648 (0.226-1.859)	0.420		
Yes		82	4				
No		304	30				
Smoking history	419			1.686 (0.772-3.682)	0.190		
Yes		75	9				
No		311	24				
Gastrointestinal bleeding				1.976 (0.887-4.401)	0.096		
Yes	422	54	8				
No		332	28				
Tumor rupture				1.810 (1.245-2.631)	0.002	1.556 (1.020-2.375)	0.040
Yes	422	62	16				
No		324	20				
Complicated with other tumors	422			0.601 (0.210-1.718)	0.342		
Yes		72	4				
No		314	32				
Tumor location	422			0.262 (0.127-0.541)	0.000	1.786 (1.261-2.5892)	< 0.001
Gastric		287	11				
No-gastric		99	25				
Tumor size (cm)	422			2.466 (1.743-3.490)	<0.001	1.693 (1.102-2.602)	0.016
≤2.0		161	2				
2.1-5.0		141	6				
5.1-10.0		59	21				
>10.0		25	7				
Mitotic count (per 50 HPFs)	415			3.208 (2.171-4.740)	<0.001	2.196 (1.421-3.392)	< 0.001
≤5		324	13				
6-10		42	7				
>10		14	15				
Ki67 (*n*%)	403			1.327 (0.606-2.906)	0.479		
<5		298	24				
>5		71	10				
Risk classification				3.865 (1.937-7.712)	<0.001	1.163 (0.527-2.568)	0.009
Low/intermediate	422	301	14				
High		85	22				

BMI: body mass index. Tumor rupture; tumor location; tumor size; mitotic count; and risk classification.

The article "Risk Factors and Prognostic Analysis of Gastrointestinal Stromal Tumor Recurrence-Metastasis" was retracted in 2023. Reasons: signs of a paper mill; suspected computer-generated content; unreliable results or conclusions; lack of ethics approval or compliance.

## Data Availability

The data used to support the findings of this study are available from the corresponding author upon request.

## References

[1] El-Menyar A., Mekkodathil A., Al-Thani H. (2017). Diagnosis and management of gastrointestinal stromal tumors: an up-to-date literature review. *Journal of Cancer Research*.

[2] Raut C. P., Morgan J. A., Ashley S. W. (2007). Current issues in gastrointestinal stromal tumors: incidence, molecular biology, and contemporary treatment of localized and advanced disease. *Current Opinion in Gastroenterology*.

[3] Søreide K., Sandvik O. M., Søreide J. A., Giljaca V., Jureckova A., Bulusu V. R. (2016). Global epidemiology of gastrointestinal stromal tumours (GIST): a systematic review of population-based cohort studies. *Cancer Epidemiology*.

[4] Ahmed M. (2020). Recent advances in the management of gastrointestinal stromal tumor. *World Journal of Clinical Cases*.

[5] Hirota S., Isozaki K., Moriyama Y. (1998). Gain-of-function mutations of c-kit in human gastrointestinal stromal tumors. *Science*.

[6] Miettinen M., Lasota J. (2003). Gastrointestinal stromal tumors (GISTs): definition, occurrence, pathology, differential diagnosis and molecular genetics. *Polish Journal of Pathology*.

[7] Joensuu H., Vehtari A., Riihimäki J. (2012). Risk of recurrence of gastrointestinal stromal tumour after surgery: an analysis of pooled population-based cohorts. *The Lancet Oncology*.

[8] Hemming M. L., Lawlor M. A., Zeid R. (2018). Gastrointestinal stromal tumor enhancers support a transcription factor network predictive of clinical outcome. *Proceedings of the National Academy of Sciences of the United States of America*.

[9] Sanchez-Hidalgo J. M., Duran-Martinez M., Molero-Payan R. (2018). Gastrointestinal stromal tumors: a multidisciplinary challenge. *World Journal of Gastroenterology*.

[10] Holmebakk T., Hompland I., Bjerkehagen B. (2018). Recurrence-free survival after resection of gastric gastrointestinal stromal tumors classified according to a strict definition of tumor rupture: a population-based study. *Annals of Surgical Oncology*.

The article "Risk Factors and Prognostic Analysis of Gastrointestinal Stromal Tumor Recurrence-Metastasis" was retracted in 2023. Reasons: signs of a paper mill; suspected computer-generated content; unreliable results or conclusions; lack of ethics approval or compliance.

[11] Vincenzi B., Nannini M., Badalamenti G. (2018). Imatinib rechallenge in patients with advanced gastrointestinal stromal tumors following progression with imatinib, sunitinib and regorafenib. *Therapeutic Advances in Medical Oncology*.

[12] Goh B. K., Chok A. Y., Allen J. C. (2016). Blood neutrophil-to-lymphocyte and platelet-to-lymphocyte ratios are independent prognostic factors for surgically resected gastrointestinal stromal tumors. *Surgery*.

[13] Miettinen M., Lasota J. (2006). Gastrointestinal stromal tumors: review on morphology, molecular pathology, prognosis, and differential diagnosis. *Archives of Pathology & Laboratory Medicine*.

[14] Kang G. H., Srivastava A., Kim Y. E. (2011). DOG1 and PKC- *θ* are useful in the diagnosis of KIT-negative gastrointestinal stromal tumors. *Modern Pathology*.

[15] Jonesuu H. (2008). Risk stratification of patients diagnosed with gastrointestinal stromal tumor. *Human Pathology*.

[16] Al-Share B., Alloghbi A., Al Hallak M. N. (2021). Gastrointestinal stromal tumor: a review of current and emerging therapies. *Cancer Metastasis Reviews*.

[17] Patel N., Benipal B. (2019). Incidence of gastrointestinal stromal tumors in the United States from 2001-2015: a United States cancer statistics analysis of 50 states. *Cureus*.

[18] Blay J. Y., Kang Y. K., Nishida T. (2021). Gastrointestinal stromal tumours. *Nature Reviews. Disease Primers*.

[19] Zhou B., Zhang M., Yan S. (2014). Primary gastrointestinal stromal tumor of the liver: report of a case. *Surgery Today*.

[20] Zemła P., Stelmach A., Jabłońska B., Gołka D., Mrowiec S. (2021). A retrospective study of postoperative outcomes in 98 patients diagnosed with gastrointestinal stromal tumor (GIST) of the upper, middle, and lower gastrointestinal tract between 2009 and 2019 at a single center in Poland. *Medical Science Monitor: International Medical Journal of Experimental and Clinical Research*.

[21] Mantese G. (2019). Gastrointestinal stromal tumor. *Current Opinion in Gastroenterology*.

[22] Kawanowa K., Skauma Y., Sakurai S. (2006). High incidence of microscopic gastrointestinal stromal tumors in the stomach. *Human Pathology*.

[23] Crosby J. A., Catton C. N., Davis A. (2001). Malignant gastrointestinal stromal tumors of the small intestine: a review of 50 cases from a prospective database. *Annals of Surgical Oncology*.

[24] Logroño R., Jones D., Faruqi S. (2004). Recent advances in cell biology, diagnosis, and therapy of gastrointestinal stromal tumor (GIST). *Cancer Biology & Therapy*.

[25] Wang Y., Peng J., Huang J. (2016). Giant and high-risk gastrointestinal stromal tumor in the abdomino-pelvic cavity: a case report. *Oncology Letters*.

The article "Risk Factors and Prognostic Analysis of Gastrointestinal Stromal Tumor Recurrence-Metastasis" was retracted in 2023. Reasons: signs of a paper mill; suspected computer-generated content; unreliable results or conclusions; lack of ethics approval or compliance.

[26] Feng F., Feng B., Liu S. (2017). Clinicopathological features and prognosis of mesenteric gastrointestinal stromal tumor: evaluation of a pooled case series. *Oncotarget*.

[27] Miettinen M., Sobin L. H., Lasota J. (2005). Gastrointestinal stromal tumors of the stomach. *The American Journal of Surgical Pathology*.

[28] Jumniensuk C., Charoenpitakchai M. (2018). Gastrointestinal stromal tumor: clinicopathological characteristics and pathologic prognostic analysis. *World Journal of Surgical. Oncology*.

[29] Liu Q. Y., Wang Y. G., Kong L. (2015). Study on clinicopathological features of gastrointestinal stromal tumor and relevant prognostic factors. *Cell Biochemistry and Biophysics*.

